# Inhibiting Cardiac Mitochondrial Fatty Acid Oxidation Attenuates Myocardial Injury in a Rat Model of Cardiac Arrest

**DOI:** 10.1155/2021/6622232

**Published:** 2021-03-01

**Authors:** Peng Wang, Fan Zhang, Liming Pan, Yunke Tan, Fengqing Song, Qiulin Ge, Zitong Huang, Lan Yao

**Affiliations:** ^1^Department of Emergency Medicine, Sun Yat-sen Memorial Hospital, Sun Yat-sen University, Guangzhou, China; ^2^Institute of Cardiopulmonary Cerebral Resuscitation, Sun Yat-sen University, Guangzhou, China; ^3^Department of Emergency Medicine, The Fifth Affiliated Hospital, Sun Yat-sen University, Zhuhai, China

## Abstract

Mitochondrial fatty acid oxidation (FAO) is involved in myocardial damage after cardiopulmonary resuscitation (CPR). This study is aimed at investigating the effect of inhibiting mitochondrial FAO on myocardial injury and the underlying mechanisms of postresuscitation myocardial dysfunction. Rats were induced, subjected to 8 min of ventricular fibrillation, and underwent 6 min of CPR. Rats with return of spontaneous circulation (ROSC) were randomly divided into the Sham group, CPR group, and CPR + Trimetazidine (TMZ) group. Rats in the CPR + TMZ group were administered TMZ (10 mg/kg) at the onset of ROSC via the right external jugular vein, while rats in the CPR group were injected with equivalent volumes of vehicle. The sham rats were only administered equivalent volumes of vehicle. We found that the activities of enzymes related to cardiac mitochondrial FAO were partly improved after ROSC. TMZ, as a reversible inhibitor of 3-ketoacyl CoA thiolase, inhibited myocardial mitochondrial FAO after ROSC. In the CPR + TMZ group, the levels of mitochondrial injury in cardiac tissue were alleviated following attenuated myocardial damage and oxidative stress after ROSC. In addition, the disorder of cardiac mitochondrial metabolism was ameliorated, and specifically, the superfluous succinate related to mitochondrial reactive oxygen species (ROS) generation was decreased by inhibiting myocardial mitochondrial FAO with TMZ administration after ROSC. In conclusion, in the early period after ROSC, inhibiting cardiac mitochondrial FAO attenuated excessive cardiac ROS generation and preserved myocardial function, probably by alleviating the dysfunction of cardiac mitochondrial metabolism in a rat model of cardiac arrest.

## 1. Introduction

Sudden cardiac arrest is a leading cause of mortality worldwide. Despite the development of cardiopulmonary resuscitation (CPR) science and the increased rate of return of spontaneous circulation (ROSC), the survival rate in patients with sudden cardiac arrest after hospital discharge remains less than 10% [1, 2]. Deaths within the first 24 h of ROSC are typically associated with multiorgan system failure, especially due to postresuscitation myocardial dysfunction [3, 4]. It is now widely believed that oxidative stress damage in the process of global myocardial ischemia/reperfusion after ROSC is the main factor linking cardiac arrest to postresuscitation myocardial dysfunction [5, 6]. Although many studies have focused on how to mitigate cardiac oxidative injury after ROSC, there remains no effective therapy for clinical application.

The generation of mitochondrial reactive oxygen species (ROS) is the main source of ROS and a crucial early driver of ischemia/reperfusion injury after ROSC [7, 8]. Uncontrolled ROS formation from the mitochondrial electron transport chain (ETC) was founded during the ischemia/reperfusion process when electrons leaking from the respiratory chain react with oxygen, especially in the hearts containing large numbers of mitochondria [9, 10]. A large body of experimental literature supports that mitochondrial ETC inhibitors appear to attenuate myocardial oxidative injury during ischemia/reperfusion [11, 12]. Our previous study found that carbon monoxide-releasing molecules decrease the generation of cardiac mitochondrial ROS and alleviate myocardial dysfunction through mildly uncoupling mitochondrial respiration in a rat model of cardiac arrest [13]. Furthermore, some studies found that excessive succinate as the substrate of mitochondrial complex II is the major source of leaking electrons and leads to extensive mitochondrial ROS formation [10, 14]. Decreasing succinate accumulation or inhibition of complex II attenuates ischemia/reperfusion oxidative injury [15]. As an intermediate substance of the citric acid cycle (CAC), succinate is affected by changes in mitochondrial metabolism. After ischemia/reperfusion, mitochondrial fatty acid and glucose utilization are damaged at different levels, while fatty acid remains the main metabolism substrate of cardiac mitochondria [16]. In some *in vitro* experiments, it was demonstrated that suppressing mitochondrial fatty acid metabolism ameliorated oxidative stress injury after ischemia/reperfusion, but the underlying mechanism is not completely deciphered [17, 18]. According to the above research results, we considered that the inhibition of mitochondrial fatty acid oxidation (FAO) may attenuate myocardial oxidative damage after ROSC by regulating mitochondrial respiratory chain substrate production, subsequently decreasing the generation of cardiac mitochondrial ROS. To investigate this, we used a rat model of cardiac arrest to examine the effect of inhibiting mitochondrial FAO on myocardial oxidative injury and the underlying mechanisms of postresuscitation myocardial dysfunction.

## 2. Materials and Methods

### 2.1. Animal Preparation and Cardiac Arrest Model

Forty-two male Sprague-Dawley rats (370-420 g) were purchased from the Medical Experimental Animal Center of Guangdong Province (Guangzhou, China). Animals were cared for in accordance with the Chinese Guidance Suggestions for the Care and Use of Laboratory Animals and with the approval of the Animal Care and Use Committee of Sun Yat-sen University.

Rats were subjected to 8 min of ventricular fibrillation (VF) and underwent 6 min of CPR. Cardiac arrest was induced by VF. Briefly, animals were anesthetized with pentobarbital sodium (45 mg/kg), and anesthesia was maintained throughout the whole experimental procedure by the additional injection of 10 mg/kg intraperitoneal pentobarbital sodium when necessary. The trachea was orally intubated with a 14-G catheter. The left femoral artery was cannulated with a polyethylene (PE) 50 catheter for blood pressure measurement. A 4F PE catheter was advanced from the right external jugular vein to the right atrium for the electrical induction of VF. During this process, cardiac rhythm and hemodynamic data were recorded using a WinDaq data acquisition system (DataQ, Akron, USA). Rectal temperature was maintained at 36.5 ± 0.5°C. After the operation, VF was induced by a 3 mA current delivered to the right ventricular endocardium through a guidewire inserted from the right external jugular vein to the right ventricle. The current flow lasted for 3 min to prevent the spontaneous reversal of VF. Following 8 min of untreated VF, the animal was mechanically ventilated (tidal volume 0.6 mL/100 g, ventilation rate 60 breaths/min, 100% oxygen), and 6 min of CPR was initiated with chest compression at a rate of 250 beats/min. After 4 min of CPR, epinephrine (0.02 mg/kg) was administered, and 3-J biphasic waveform shocks were attempted after 6 min of CPR. If VF persisted, another 3-J shock was administered after another 2 min of chest compression. Successful ROSC was defined as an organized rhythm with a mean aortic pressure (MAP) exceeding 60 mmHg for at least 10 min. If the animals had no ROSC after 10 min of CPR, unsuccessful resuscitation was declared. After ROSC, mechanical ventilation was continuously provided with 100% oxygen for 30 min and 50% oxygen for another 30 min, followed by 21% oxygen for 3 h.

### 2.2. Experimental Procedure

Trimetazidine (TMZ), a reversible inhibitor of 3-ketoacyl CoA thiolase (3-KT), was used to inhibit cardiac mitochondrial FAO. A total of 36 rats with successful ROSC were randomly divided into the CPR (*n* = 18) and CPR + TMZ (*n* = 18) groups. Rats in the CPR + TMZ group were administered TMZ (MedChemExpress, USA; 10 mg/kg, 10% dimethyl sulfoxide as a vehicle) at the onset of ROSC via the right external jugular vein, while those in the CPR group were injected with equivalent volumes of vehicle. The sham rats (*n* = 6) were only administered equivalent volumes of vehicle. Rats in the CPR and CPR + TMZ groups were again randomly divided into three subgroups according to the time of ROSC (1, 3, and 6 h after ROSC). Myocardial injury, oxidative stress, and cardiac mitochondrial metabolism and function were evaluated. The experimental procedure is shown in Figure 1.

### 2.3. Measurement of Serum Cardiac Troponin I and Myocardial Function

Cardiac troponin I (CTNI) levels in serum were detected using a Rat CTNI ELISA kit (CUSABIO, China). An M-mode echocardiograph was performed to detect the left ventricular ejection fraction (EF) to evaluate myocardial function.

### 2.4. Determination of Malondialdehyde in Myocardial Tissue and Cardiac Mitochondrial ROS

Malondialdehyde (MDA) is an evaluation indicator of oxidative stress indicators. The level of MDA in myocardial tissue was measured using a tissue MDA determination kit (GENMED, Boston, MA, USA). Cardiac mitochondria were isolated by differential centrifugation of the heart homogenates. Fresh cardiac mitochondria were loaded with a reagent containing the fluorescent probe (CM-H_2_DCFDA) for 15 min. Fluorescence was measured using a fluorescence spectrophotometric enzyme mark instrument (SpectraMax M5, San Francisco, CA, USA) following the manufacturer's instructions for the mitochondrial ROS testing kit (GENMED).

### 2.5. Measurement of Mitochondrial Oxidative Phosphorylation and Respiration Enzyme Activities

The mitochondrial P/O ratio was used to evaluate the coupling of mitochondrial oxidative phosphorylation by a Clark-type oxygen electrode at 25°C. Fresh cardiac mitochondria were added to the respiration buffer (GENMED, Boston, MA, USA). Mitochondrial respiration was initiated using 2 mmol/L pyruvate +5 mmol/L malate. State 3 respiration was induced by the addition of 0.5 mmol/L adenosine diphosphate (ADP). The ADP to O ratio was calculated based on the oxygen consumption during state 3 respiration. The activities of complexes I and II were measured using a mitochondrial respiratory enzyme activity determination Kit (GENMED, Boston, MA, USA). Complex I and II activities were assayed to monitor the dynamic change in transmittance from the oxidation of NADH to NAD^+^ and FADH_2_ to FAD^+^.

### 2.6. Detection of FAO-Related Enzyme Activities

Isolated mitochondria from the heart were suspended in 24-well plates. The rate of mitochondrial FAO was evaluated by using a fatty acid *β*-oxidation Assay kit (GENMED, Boston, Massachusetts). The activities of carnitine palmitoyltransferase 1 (CPT1), acyl-CoA dehydrogenase (ACDH), 3-OH-ACDH (HADH), and 3-KT as important enzymes in mitochondrial FAO were measured using their respective commercial enzyme activity determination kits (GENMED, Boston, Massachusetts).

### 2.7. Metabolite Analysis

Sample preparations for targeted GC-MS metabonomic analysis were established as previously reported [19]. Then, 30 mg of left ventricle tissue from each mouse in the sham, CPR, and CPR + TMZ groups at 6 h of ROSC was mixed with 1 mL of methanol and ultrasonically ground for 30 min. The supernatant was then added to 2 mL of 1% sulfuric acid methanol solution. After methylation for 30 min at 80°C, the mixture was extracted with 1% hexane and washed with 5 mL of pure water. The supernatant (500 *μ*L) was then collected for GC-MS metabolomics analysis. In parallel, 37 kinds of fatty acid methyl ester standards were proportionally mixed as the standard for target analysis of medium- and long-chain fatty acids. A quality control (QC) sample was prepared by mixing equal volumes (10 *μ*L) of ventricle homogenate from each of the 18 samples. One in every six QC samples were analyzed to monitor the stability and reproducibility of the analysis. The samples were separated using an Agilent DB-WAX capillary column (30 m × 0.25 mM × 0.25 *μ*M). The initial temperature of the capillary column was maintained at 50°C for 3 min, raised to 220°C at 10°C/min, and then kept at this temperature for 20 min. The carrier gas (helium) was constantly supplied at a flow rate of 1.0 mL/min. GC-MS analysis was carried out using an Agilent 7890a/5975c gas chromatography mass spectrometer (Agilent, USA). The temperature of sample inlet, transmission line, and ion source temperature were 280°C, 250°C, and 230°C, respectively. The electron energy was set to 70 eV. The peak area and retention time data were extracted using the MSD ChemStation software. The levels of targeted medium- and long-chain fatty acids were calculated according to the total ion current picture of fatty acid standards.

To detect the content of metabolites mainly in CAC and glycolysis by targeted GC-MS metabolomic analysis, the samples were separated using an Agilent 1290 infinity liquid chromatography ultraperformance system. A QC sample from the experimental samples at each interval was established to detect and evaluate the stability and repeatability of the system. A standard mixture of substances from the sample queue was used to correct the chromatographic retention time. The samples were analyzed using a 5500 qtrap mass spectrometer (AB SCIEX) in negative ion mode. The detection settings were as follows: source temperature 450°C, ion source gas 145, ion source gas 245, culture gas 30, and floating voltage -4500 V. The MRM mode was used to detect ion pairs. Metabolite identification and retention time correction were performed according to the data of the standard mixture of substances. The peak area and retention time were extracted and calculated using the MultiQuant software.

The levels of free fatty acids (FFAs) and glucose in serum were estimated using an FFA Quantification Colorimetric/Fluorometric Kit (BioVision, Milpitas, CA, USA) and a Rat Glucose Quantification Kit (CUSABIO).

### 2.8. Pathological Examination of Myocardial Tissue

Left ventricular tissue was embedded in paraffin and cut into 6 *μ*M thick sections following hematoxylin and eosin staining. Myocytolysis and organization of myocardial fibers were observed under a microscope by an experienced pathologist.

### 2.9. Transmission Electron Microscopy

Apex tissue (3 × 1 × 1 mM) was prefixed in 2.5% glutaraldehyde and then added to 1% osmium tetroxide for continuous fixation and dehydrated in a gradient concentration of acetone series. After infiltration and embedding, the sample was sliced into ultrathin sections stained with both uranyl acetate and lead citrate. Samples were examined using a transmission electron microscope (Tecnai G2 Spirit Twin, FEI, USA).

### 2.10. Statistical Analysis

Statistical analyses were performed using the SPSS 21.0 software (SPSS, Chicago, IL, USA). Data are presented as the mean ± SEM. One-way analysis of variance was performed to compare more than two groups. The unpaired two-sample *t*-test was used for two-group comparison. Values of *p* < 0.05 were considered statistically significant.

## 3. Results

### 3.1. Baseline Characteristics and Hemodynamic Data before Inducing Cardiac Arrest

A total of 36 successfully resuscitated rats were randomly assigned to the Sham, CPR, or CPR + TMZ groups. The baseline and resuscitation characteristics of the rats were recorded. There was no significant difference in body weight, heart rate, MAP, or time of animal preparation in any group (Table 1).

### 3.2. TMZ Inhibited Myocardial Mitochondrial FAO after ROSC

The activities of enzymes related to mitochondrial FAO were evaluated in the heart. 1 h after ROSC, the activities of 3-KT (Figure 2(a)), CPT1 (Figure 2(b)), and ACDH (Figure 2(c)) were markedly elevated compared with the Sham group. Additionally, 3 h after ROSC, the activity of CPT1 (Figure 2(b)) remained higher, but there was no significant difference in the activities of 3-KT and ACDH (Figures 2(a) and 2(c)). Although the CPR group exhibited slightly increased activity of each related enzyme 6 h after resuscitation, there were no statistically significant differences between the sham and CPR groups. The activity of HADH (Figure 2(d)) did not obviously change after ROSC. In the TMZ group, TMZ, a reversible inhibitor of 3-KT, remarkably decreased the activity of 3-KT (Figure 2(a)) in the heart after ROSC compared with the CPR group. Meanwhile, the administration of TMZ evidently decreased the activity of CPT1 (Figure 2(b)) at 3 h and increased the activity of HADH (Figure 2(d)) in the heart at 6 h following ROSC, leading to the enzymatic activity being nearly restored to the levels of the Sham group. Together, these observations indicated that myocardial energy metabolism was abnormally mobilized, and myocardial mitochondrial FAO was relatively accelerated after ROSC. TMZ effectively inhibited myocardial mitochondrial FAO during the early stage of ROSC due to the decrease in some key enzyme activities.

### 3.3. Inhibition of Mitochondrial FAO Attenuated Myocardial Injury after ROSC

After cardiac arrest, the levels of CTNI (Figure 3(a)) were significantly higher than those in the sham group. Rats in the CPR group showed a decrease in MAP (Figure 3(b)) and EF (Figure 3(c)) compared with sham rats. At 1, 3, and 6 h after ROSC, TMZ reduced the content of CTNI (Figure 3(a)) in blood serum as well as elevated MAP (Figure 3(b)) and EF (Figures 3(c) and 3(d)) in the CPR + TMZ group compared with the CPR group. At 6 h following ROSC, myocytolysis and disorganization occurred in the CPR group (Figure 3(e)). The ROSC rats treated with TMZ significantly alleviated myocytolysis and disordered myocardial fibers in the CPR + TMZ group (Figure 3(e)). These findings revealed that inhibition of mitochondrial FAO mitigated myocardial injury and improved myocardial performance after resuscitation.

### 3.4. Inhibition of Mitochondrial FAO Decreased Myocardial Oxidative Stress after ROSC

Cardiac mitochondria, as the main site of energy production, are also the main source of ROS after cardiac arrest. In the CPR group, the generation of ROS in cardiac mitochondria significantly increased 1 and 6 h after ROSC compared with the Sham group (Figure 4(a)). However, TMZ led to less ROS production in cardiac mitochondria in the CPR + TMZ group than in the CPR group (Figure 4(a)). Moreover, the levels of MDA in the CPR group were significantly higher than those in the sham group (Figure 4(b)). Moreover, 1, 3, and 6 h after ROSC, TMZ reduced the content of MDA in the heart (Figure 4(b)).

### 3.5. Inhibition of Mitochondrial FAO Preserved Mitochondrial Function after ROSC

To further evaluate the coupling of mitochondrial oxidative phosphorylation and the activities of respiratory enzymes related to mitochondrial ROS production, the ADP/O ratio and the activities of complexes *Ι* and II were detected. First, 1 and 6 h following ROSC, the ADP/O of cardiac mitochondria in the CPR group was markedly decreased compared with those of the Sham group (Figure 5(a)). Inhibition of mitochondrial FAO with TMZ treatment improved ADP/O after ROSC in the TMZ group (Figure 5(a)). Meanwhile, there was a significant decline in the activities of complexes I and II 1 and 6 h after ROSC (Figures 5(b) and 5(c)). In the TMZ group, TMZ significantly alleviated the damage to complex I (Figure 5(b)) and complex II activities (Figure 5(c)) after ROSC. Transmission electron microscopy showed cardiac mitochondrial morphology in the CPR group was represented as mitochondrial swelling and unclear intima 6 h after ROSC (Figure 5(d)). Inhibition of mitochondrial FAO in the CPR + TMZ group obviously mitigated cardiac mitochondrial injury in the electron microscope image compared with the CPR group (Figure 5(d)).

### 3.6. Inhibition of Mitochondrial FAO Ameliorated the Disorder of Cardiac Mitochondrial Metabolism after ROSC

We found that the concentrations of FFAs (Figure 6(a)) and glucose (Figure 6(b)) in serum significantly increased after ROSC. TMZ treatment decreased FFA (Figure 6(a)) and glucose (Figure 6(b)) levels compared with CPR rats. Targeted metabolomics analysis of medium- and long-chain fatty acids and energy metabolites in heart tissue was carried out 6 h after ROSC. We found that the levels of five fatty acids were evidently decreased, while four metabolites were upregulated significantly in the heart tissue of CPR rats compared with that of sham rats. The lengths of the five decreased fatty acids were in the range of C12-C22, closely related to mitochondrial FAO. Three elevated metabolites (succinate, fumarate, and citrate) were the main intermediate products of CAC, and succinate was the substrate of the ETC bound to mitochondrial ROS generation. Elevated phosphoenolpyruvate was the main metabolite of glycolysis. In the TMZ group, these changed metabolites were normalized to some extent through the inhibition of mitochondrial FAO (Table 2). These results showed that inhibiting mitochondrial FAO after ROSC restored the balance of cardiac mitochondrial metabolism.

## 4. Discussion

In this study, we showed that the inhibition of myocardial mitochondrial FAO attenuates myocardial injury and protects cardiac mitochondrial function after ROSC. The underlying mechanism is that FAO inhibition in cardiac mitochondria ameliorates the mitochondrial metabolism disorder and abnormal generation of ETC substrates, subsequently leading to the decrease in excessive ROS production in cardiac mitochondria after ROSC. Several findings in the present study support this conclusion. First, we found that the activities of some key FAO enzymes in cardiac mitochondria were elevated, and the levels of fatty acids in serum were markedly increased at the early stage of ROSC. 3-KT inhibitor TMZ repressed abnormal FAO in cardiac mitochondria and improved myocardial performance in ROSC rats. These results indicated that the suppression of activated FAO attenuated postresuscitation injury in the heart. Second, the excessive production of cardiac mitochondrial ROS significantly decreased following treatment with TMZ after ROSC. The alleviation of mitochondrial dysfunction was also found in the CPR + TMZ group. These findings demonstrated that the inhibition of cardiac FAO decreased mitochondrial ROS generation to mitigate cardiac oxidative injury and protected mitochondrial function after ROSC. Third, the anomalous level of succinate as an important ETC substrate in heart tissue, which is evidently related to excessive mitochondrial ROS generation, was reduced after ROSC with TMZ treatment. The abnormalities of fatty acid metabolism in cardiac mitochondria after cardiac arrest were reversed to some extent by the inhibitor TMZ. Simultaneously, the injury of glycometabolism in cardiac mitochondria was mitigated. These results indicated that the inhibition of FAO at the early stage of ROSC decreased mitochondrial ROS generation by reduction of abnormal mitochondrial metabolites. Several previous studies have demonstrated that inhibition of myocardial FAO attenuates ischemia/reperfusion injury by affecting AMPK and ERK signaling pathways, activating pyruvate dehydrogenase, and so on [17, 20]. However, there have been no studies involving to the effects of FAO inhibition on abnormal ROS generation in the cardiac mitochondria of cardiac arrest models and the underlying mechanism. Thus, this study showed that inhibition of myocardial FAO in the early stage of ROSC attenuates excessive ROS generation in cardiac mitochondria by decreasing the levels of abnormal mitochondrial substrates and modulating mitochondrial metabolism, leading to the mitigation of myocardial injury after ROSC.

In the normal heart, cardiac mitochondria are the main source of energy supply, and fatty acid *β*-oxidation is responsible for 60-80% of ATP production [3, 21]. After ischemia/reperfusion, although impaired mitochondrial oxidative phosphorylation results in a decline in ATP supply, fatty acid *β*-oxidation remains the dominant process of mitochondrial oxidative metabolism due to compensatory catecholamine discharge, accelerated adipose tissue lipolysis, increased plasma concentrations of FFA, etc. [16, 22]. Similar to the results of previous studies, we identified elevated activities of CPT1, 3-KT, and ACDH as the key enzymes of FAO in the heart tissue and increased levels of FFAs in ROSC rats. This suggests that fatty acid *β*-oxidation plays an important role in cardiac mitochondrial metabolism after ROSC. To further determine the effect of *β*-oxidation, we used a reversible 3-KT inhibitor, TMZ, to intervene in fatty acid *β*-oxidation at the early stage of ROSC. In the CPR + TMZ group, TMZ not only decreased the activities of 3-KT and CPT1 as well as FFA levels after ROSC but also mitigated cardiac dysfunction and myocardial injury in cardiac arrest rat models. Strong evidence of this lay in improved EF and MAP following a reduced concentration of CTNI compared with the CPR group. The reduction of FAA in TMZ group may result from gradually rebalanced metabolism and reduced compensation of adipose tissue lipolysis after ROSC [21]. Furthermore, the MDA content of cardiac tissue was markedly lower in the CPR + TMZ group. It was known that oxidative injury is one of the most important pathological mechanisms in myocardial damage after ROSC [23, 24]. These results indicated that the inhibition of fatty acid *β*-oxidation attenuates myocardial oxidative damage to preserve cardiac function after ROSC. The consistent viewpoint was found in some researches on heart failure, myocardial hypertrophy, etc. [25].

Cardiac mitochondria, the main site of ATP production, are also the major source of ROS in the hearts subjected to ischemia/reperfusion injury [23]. Moreover, excessive ROS leads to cardiac mitochondrial dysfunction, which results in increased ROS generation in cardiac mitochondria and decreased ATP generation, forming a vicious cycle [26]. Several recent studies showed that mitochondrial ROS generation in pathological conditions is closely related to the disorder of mitochondrial metabolism [25, 27]. In our study, rats in the CPR + TMZ group showed elevated ADP/O of cardiac mitochondria and partial restoration of complex *Ι* and II activities compared with the CPR group. It was known that complexes *Ι* and II are the main sites of ETC accepting electrons to form ATP and ROS both in normal and pathological conditions [10, 27]. Attenuation of complex *Ι* and II damages led to a decrease in excessive ROS generation in cardiac mitochondria, probably due to less electron leakage and increased ATP production in ROSC rats with TMZ treatment. These findings showed that the inhibition of fatty acid *β*-oxidation mitigated excessive ROS generation in cardiac mitochondria and preserved their function, resulting in the attenuation of myocardial oxidative stress after cardiac arrest in a rat model. Previous studies supported abnormal ROS production in cardiac mitochondria plays an important role in oxidative injury in pathological conditions [26, 28]. It is well known that the excessive ROS generation is caused by the abnormal electron leak of the ETC related to mitochondrial dysfunction and aberrant metabolism in the pathological state of myocardia [29].

In this study, we found that the concentration of succinate, as the substrate of complex II, increased 6 h after ROSC in cardiac tissue, with an improved level of its subsequent metabolite fumarate in CAC. These observations indicate that superfluous succinate mismatches the acceptance of injured mitochondria in cardiac tissue, resulting in ETC electron leak and excessive ROS production after ROSC [11, 14]. In view of CAC metabolites mainly stemming from mitochondrial fatty acids and glucose metabolism, the levels of other metabolites and some key enzymes were also detected. In the hearts of CPR rats, it was found that the content of five fatty acids (C12-C22) decreased, while phosphoenolpyruvate as the intermediate of glycolysis increased significantly 6 h after ROSC. In addition, the key enzyme activities of FAO, including CPT1, ACDH, and 3-KT, were elevated during the early postresuscitation period. These results prompted the hypothesis that excessive succinate formation in the heart after ROSC is related to comparatively elevated FAO. Some previous researches showed that partial inhibition of FAO mitigates the damage of cardiac cells and mitochondria in some pathological conditions, although the underlying mechanism is currently unclear [25]. To investigate the effect of elevated cardiac FAO in CPR rats, we used TMZ to suppress FAO and detected mitochondrial metabolism after ROSC. In the CPR + TMZ group, we found that the levels of succinate and fumarate were reduced while the content of five fatty acids increased with the alleviation of ROS injury in cardiac tissue 6 h after ROSC. Moreover, the level of phosphoenolpyruvate simultaneously decreased to that of the Sham group. These findings indicated that the inhibition of abnormal FAO prompted the optimization of impaired mitochondrial metabolism and mitigated ROS injury in cardiac tissue during the early stage of ROSC, potentially due to the decrease of unsuitable ETC substrates offering excessive electrons to form ROS. Some studies also supported that the reduction of abnormal succinate may decrease ROS generation in ischemia-reperfusion injury [14, 30].

There are still some limitations in the current study. First, we only investigated the relationship between abnormal mitochondrial metabolism and excessive ROS production in the early stages of ROSC. Regarding postresuscitation cardiac damage and oxidative injury lasting several days, the long-term effect of abnormal FAO on cardiac oxidative stress requires determination. Second, in our study, we focused on the effect of abnormal FAO on unsuitable mitochondrial FAO and glycolysis metabolites and superfluous ROS generation in cardiac mitochondria after ROSC in rats. Other pathways of cardiac mitochondrial metabolism, such as amino acid metabolism, have not been studied.

## 5. Conclusion

The inhibition of cardiac mitochondrial FAO mitigates abnormal cardiac ROS production and myocardial injury as well as effectively improves cardiac function, in part, by alleviating the mitochondrial metabolism disorder and uncoupled mitochondrial oxidative phosphorylation in a rat model of cardiac arrest.

## Figures and Tables

**Figure 1:** Experimental procedure. CPR: cardiopulmonary resuscitation; TMZ: trimetazidine; FFA: free fat acid; GLU: glucose; ROSC: return of spontaneous circulation; mitROS: mitochondrial reactive oxygen species; TEM: transmission electron microscope.

**Figure 2:** The enzyme activities of mitochondrial fatty acid oxidation in rat heart tissue at 1, 3, and 6 h following return of spontaneous circulation (ROSC) in the CPR and CPR+ Trimetazidine (TMZ) groups compared with the Sham group: (a) 3-ketoacyl CoA thiolase (3-KT) activity; (b) carnitine palmitoyltransferase 1 (CPT1) activity; (c) acyl-CoA dehydrogenase (ACDH) activity; (d) 3-OH-acyl CoA dehydrogenase (HADH) activity. *^β^p* < 0.05, ^∗^*p* < 0.01 versus Sham group; ^#^*p* < 0.05, ^$^*p* < 0.01 versus CPR group.

**Figure 3:** Myocardial injury at 1, 3, and 6 hours following return of spontaneous circulation (ROSC) in the CPR and CPR + Trimetazidine (TMZ) groups compared with the Sham group: (a) cardiac troponin I (CTNI); (b) mean aortic pressure (MAP); (c) left ventricular ejection fraction (EF); (d) representative echocardiograms in three groups at 6 hours following ROSC; (e) pathological examination of myocardial tissue in three groups at 6 hours following ROSC. Magnification ×200. *^β^p* < 0.05, ^∗^*p* < 0.01 versus Sham group; ^#^*p* < 0.05, ^$^*p* < 0.01 versus CPR group.

**Figure 4:** Cardiac mitochondrial oxidative stress at 1 and 3 hours following return of spontaneous circulation (ROSC) in the CPR and CPR + Trimetazidine (TMZ) groups compared with the Sham group: (a) cardiac mitochondrial reactive oxygen species (ROS); (b) malondialdehyde (MDA). ^∗^*p* < 0.01 versus Sham group; ^$^*p* < 0.01 versus CPR group.

**Figure 5:** Cardiac mitochondrial function at 1 and 3 hours following return of spontaneous circulation (ROSC) in the CPR and CPR + Trimetazidine (TMZ) groups compared with the Sham group: (a) ADP/O ratio; (b) mitochondrial complex I activity; (c) mitochondrial complex II activity; (d) representative transmission electron microscope images of cardiac mitochondria at 6 hours following ROSC. *^β^p* < 0.05, ^∗^*p* < 0.01 versus Sham group; ^#^*p* < 0.05, ^$^*p* < 0.01 versus CPR group.

**Figure 6:** The levels of free fat acid and glucose in serum at 1, 3, and 6 hours following return of spontaneous circulation (ROSC) in the CPR and CPR + TMZ groups compared with the Sham group: (a) the level of free fat acid; (b) the level of glucose. *^β^p* < 0.05, ^∗^*p* < 0.01 versus Sham group; ^#^*p* < 0.05, ^$^*p* < 0.01 versus CPR group.

**Table 1:** Baseline characteristics before inducing cardiac arrest.

	Sham	CPR groups			CPR + TMZ groups		
		1 h	3 h	6 h	1 h	3 h	6 h
Body weight, g	392.3 ± 14.7	386.8 ± 14.8	392.3 ± 21.2	395.7 ± 16.3	394.7 ± 12.9	390.3 ± 15.1	393.2 ± 14.9
MAP, mmHg	110.3 ± 9.8	114.5 ± 11.5	111.2 ± 11.1	111.8 ± 10.1	112.5 ± 9.8	107.3 ± 11.3	108.2 ± 15.5
Heart rate, bpm	392.7 ± 11.4	395.0 ± 9.4	392.7 ± 11.5	393.3 ± 11.2	394.2 ± 7.4	393.0 ± 11.9	391.8 ± 12.2
Time of animal preparation, min	61.8 ± 5.4	63.7 ± 7.3	65.3 ± 6.0	62.7 ± 8.5	57.0 ± 6.4	61.8 ± 7.5	60.7 ± 9.7

**Table 2:** The change of cardiac mitochondrial metabolites at 6 hours following return of spontaneous circulation.

Mitochondrial metabolites	Sham group	CPR group	CPR + TMZ group
Lauric acid (*μ*g/g)	0.56 ± 0.13	0.05 ± 0.03^∗^	0.33 ± 0.15^∗^^,$^
Myristic acid (*μ*g/g)	23.54 ± 10.58	7.29 ± 0.98^∗^	17.58 ± 2.44^#^
Palmitoleic acid (*μ*g/g)	81.54 ± 31.97	25.98 ± 9.47^∗^	53.15 ± 13.35^*β*,#^
Elaidic acid (*μ*g/g)	1245.51 ± 302.98	394.61 ± 55.86^∗^	779.61 ± 219.82^∗^^,$^
Docosadienoic acid (*μ*g/g)	3.22 ± 0.85	1.28 ± 0.52^∗^	2.96 ± 0.78^$^
Succinate (AU)	97601.71 ± 12955.30	131530.6593 ± 16054.71^∗^	103200.39 ± 10078.42^$^
Phosphoenolpyruvate (AU)	9510787.49 ± 5590095.37	21573980.98 ± 5517056.59^∗^	15001059.54 ± 2808820.31^#^
Fumarate (AU)	865263.39 ± 210253.45	2111186.90 ± 627354.51^∗^	1565341.13 ± 290282.39^*β*,#^
Citrate (AU)	111084.32 ± 16644.73	179985.21 ± 32520.83^∗^	114157.36 ± 38654.61^$^

Values are means ± SE; *^β^p* < 0.05, ^∗^*p* < 0.01 versus Sham group; ^#^*p* < 0.05, ^$^*p* < 0.01 versus CPR group.

## Data Availability

The data used to support the findings of this study are available from the corresponding author upon request.
